# Extent of COVID-19 Healthcare Services of Isolation Center of Private Hospital across Khartoum State, Sudan

**DOI:** 10.1155/2022/6745813

**Published:** 2022-03-23

**Authors:** Ghada Omer Hamad Abd El-Raheem, Maysoun Ahmed Awad Yousif, Doaa Salih Ibrahim Mohamed, Ragaa Omer Gasmelsaid Farah, Mohamed Elfatih Abdalla Bukhari, Nehal Faysal Ezalden Mohamed, Mohammednour Omer Ahmad, Braa Kamal Ismail Saeed

**Affiliations:** ^1^Pharmacy Department, Imperial Specialized Hospital, Alsharif Alhindi Street, Khartoum, Sudan; ^2^Emergency Department, Imperial Specialized Hospital, Alsharif Alhindi Street, Khartoum, Sudan

## Abstract

**Introduction:**

Spatial presentation is considered a useful tool for analyzing and mapping the frequencies of incidences of different pathogens. Khartoum State accounted for 78% of the overall cases of COVID-19 in Sudan. The aim of this study was to present the spatial extent of healthcare services of a private isolation center during the pandemic at the locality level.

**Materials and Methods:**

A spatial descriptive study was conducted using ArcGIS to present the locations of all COVID-19 patients who attended Imperial Hospital isolation center on November–December 2020 in Khartoum, Sudan.

**Results:**

Patients diagnosed with COVID-19 during the study period were 188; they had attended Imperial Hospital from 9 states. Patients from Khartoum State were 167 patients. Of those 167 patients, 75 were from the Khartoum locality; it is the locality in which Imperial Hospital is located, followed by Khartoum Bahri (34 patients), Omdurman (19 patients), and South Khartoum (14 patients), while 10 patients each were from the Sharg En Nile and Karary localities.

**Conclusion:**

Patients from 8 different states of Sudan had travelled to reach Khartoum State to get health services. At the state level, Khartoum State was the most benefited state from the healthcare services of Imperial Hospital. At a locality level, Khartoum locality was the most benefited one.

## 1. Introduction

Coronavirus 19 (COVID-19) is an emergent global health situation; it was declared a pandemic by the WHO [1]. Even though this virus might cause mild disease in many people, the course of infection and illness might be severe, leading to hospitalization and even death among the elderly population or those with comorbid conditions [2]. The global spread of the COVID-19 pandemic led to massive socioeconomic and health issues across the whole world. This pandemic continues to gallop worldwide, and this situation tests the capacity of hospitals and the strength of healthcare systems [3]. The spatial presentation has been considered as a useful tool for analyzing spatial epidemiology through mapping and analyses of spatial and spatial-temporal frequencies of incidences of different pathogens [4]. Spatial-based techniques are used to properly understand and investigate outbreaks. As well as, analyze the epidemiological risks providing a relevant tool for healthcare management [5]. Based on the low healthcare capacity, identification of high-risk areas is a logical step for developing more effective strategies to mitigate the risk where the more susceptible populations are located [5, 6]. The most important features of pandemics are spatial dissemination and transmission. Those features depend mainly on spreading mechanisms, human mobilization, and pandemic control strategies [7]. To properly understand the complete dynamics of this pandemic, we need a subnational level data analysis; this allows us to account for the geographical variations between different populations for the provision of healthcare services [8]. Poor public health foundation is the main limitation and disadvantage in the strategies against the COVID-19 pandemic. It increases the risk of spread [9]. As per United Nations reports, Khartoum State accounted for 78% of the overall COVID-19 cases in Sudan [10].

The aim of this study was to present the spatial extent of healthcare services during the COVID-19 pandemic to assess the capacity of health coverage at the locality level. The rationale of this study during the ongoing pandemic was to present the spatial extent of healthcare services of an isolation center in Khartoum State. This spatial presentation is helpful for Sudan as it provided the areas covered with the medical care of COVID-19 patients during the pandemic. This will help concerned authorities identify the spatial gaps in healthcare services.

## 2. Materials and Methods

A descriptive study was conducted to record the residences and locations of all COVID-19 patients who attended Imperial Hospital isolation center in November and December 2020 in Khartoum State, Sudan. Imperial Hospital is a 60-bed hospital. It contains three isolation wards as well as an isolation emergency room. General isolation wards were a 2 with 10 bed capacity each, while the isolation ICU had a 5 bed capacity. Patients with suspected COVID-19 infection were admitted and quarantined in this tertiary care hospital. Nasal swabs were collected and tested for the presence of SARS-CoV-2 through the reverse transcriptase-polymerase chain reaction (RT-PCR) test. Once patients were confirmed as COVID-19 positive by the RT-PCR, they were shifted to the isolation ward. 188 patients who attended in November 2020 and December 2020 were involved in the study. The locations of the residences were requested from the patients and recorded. Patients gave their assent to provide their residences for this paper. The geographic information system (GIS) ArcGIS 10.3 was used to develop the maps at two levels; the state level and the localities of Khartoum State level. Data were entered as attribute tables to the ArcMap program. Microsoft Excel and the Statistical Package of Social Sciences (SPSS-23) were used in the data entry process. Longitude (LON) and latitude (LAT) coordinates of the states of Sudan and the localities of Khartoum State were used to present the locations in the thematic maps. Prevalence was calculated as cases per 10,000 populations. The kriging method was used to develop the risk map. A hotspot analysis was conducted to determine the clustered areas in the localities of Khartoum State. As well, the radius of the area covered by Imperial Hospital services was obtained through ArcMap.

## 3. Results

### 3.1. Healthcare Services of Imperial Hospital for COVID-19 Patients across the States of Sudan

Imperial Hospital is a private tertiary hospital with isolation centers for COVID-19 patients. It is located in Khartoum city, Khartoum State. 188 patients attended Imperial Hospital during the second wave of the COVID-19 pandemic in November and December 2020. Those patients came to Imperial Hospital from 9 states of Sudan. The majority of the cases, 167 cases, were from Khartoum State, followed by Northern and El Gezira states, 8 and 4, respectively. The rest of the states had lower frequencies of patients (Figure 1). States and case distribution are described in Figure 1.

### 3.2. Healthcare Services of Imperial Hospital for COVID-19 Patients across the Localities of Khartoum State

There were 167 patients who attended Imperial Hospital which is located in Khartoum State. Khartoum State is comprised of 7 localities. Of the 167 patients, 75 were located in the Khartoum locality. In this locality, Imperial Hospital is located, followed by Khartoum Bahri locality, from which 34 patients have received COVID-19 care at Imperial Hospital. 19 patients were located in the Omdurman locality. 14 patients were located in the South Khartoum locality. On the other hand, 10 patients from Sharg En Nile and Karary localities each had reached for COVID-19 care in Imperial Hospital. The least number of patients were from Um Badda locality (5 patients).  Figure 2 shows the thematic map describing the extent of healthcare services across the State of Khartoum.

On hotspot analysis of Khartoum State, the highest clustered area was Khartoum locality. Other localities were not significant for any clusters, Figure 3.

The population of Khartoum State per each locality was estimated for the year 2020 in Figure 3. Um Badda and South Khartoum were the most habituated localities, followed by Shrag En Nile and Khartoum localities. Of those 4 highly habituated localities, Khartoum locality is the smallest in size. Most cases of COVID-19 were from the Khartoum locality, as it is the locality in which Imperial Hospital is located.  Figure 4 illustrates the habitants and the cases at each locality in Khartoum State.

### 3.3. Radius of Imperial Healthcare Services for COVID-19 Patients across Khartoum State

The radius of Imperial Hospital Healthcare Services for COVID-19 patients was detected through buffer analysis. The 204 km radius was the extension of healthcare services for COVID-19 cases across Khartoum State localities.  Figure 5 illustrates the radius of COVID-19 services provided by Imperial Hospital.

The risk map in Figure 4 illustrates the prediction of COVID-19 infection across the state of Khartoum. All the state localities had the prevalence calculated as cases per 10000 population (Figure 6)

## 4. Discussion

Although Imperial Hospital is considered a small hospital, the extent of healthcare services has reached the state-level. Besides Khartoum State, other 8 states had benefited from the services of the isolation center of Imperial hospital. 88% of the cases were from Khartoum State; this might be related to the fact that Imperial Hospital is located in Khartoum, as well as reports have indicated that the majority of COVID-19 cases were located in Khartoum State [10]. We assessed the population density in each locality as the density of habitants was considered an important factor for COVID-19 risk [1]. In Khartoum State, all 7 localities were covered by the healthcare services of Imperial Hospital. Khartoum locality had a high density of habitats compared to its size, as highly populated areas particularly face high pandemic risks [7]. Urbanization involves the heavy habitation of populations in the cities [7]. That was the case with Khartoum locality in particular and Khartoum State in general. The Khartoum locality was the most benefited locality. This can be explained by the ease of accessibility to the hospital, as Imperial Hospital is located in this locality. Reaching out for healthcare services from distant areas has been a suffering issue, not only in Sudan but in India as well [9]. Some studies were concerned with nation-wide and state-level spatial analysis [1, 6, 11], and other spatial studies presented their data at the provenance level [4, 8] as well as the district level [9]. Our study presented results at localities of Khartoum State, in a spatial presentation, unlike studies [1, 11] which were concerned with state-level COVID-19 risk. This study is similar in aspect to an Indian study of a tertiary hospital in Pune city, India, describing the spread of 197 cases across the city [2]. Besides the COVID-19 healthcare extension, this study showed wide variations in the number of populations across different localities. Some localities, such as Um Badda, Khartoum, and South Khartoum, had high populations compared to their sizes. While others such as Khartoum Bahri had a low population compared to the size of the locality. These variations between sizes and densities of inhabitants have been reported in the provenances of Iran [4]. Prediction of the area at risk was presented as a risk map through the kriging method, while another study identified high-risk areas through bivariate maps describing ICU cases and mortality risk [6]. Here in Sudan, private hospitals had the equivalent capacity to receive COVID-19 patients and provide both inpatient and outpatient healthcare services; even home oxygen was provided by the hospital pharmacy for outpatients and discharged patients who had a moderate infection. Similar to governmental isolation centers, medications were also provided in addition to oxygen. Our study spatially described COVID-19 healthcare, while, in another study, COVID-19 mortality was described [8]. Alarmingly, our study showed that COVID-19 patients had to travel from 8 different states to reach Khartoum State to receive health services.

The limitations of our study were the enrolment of a single-center for healthcare assessment. Moreover, the governmental section was not covered in this study. Another limitation was the low possibility of generalization of the results to other countries. Follow-up of patients for their outcome was not part of the objectives of this study. However, our results can be used as a part of the baseline data for assessing healthcare system coverage in Sudan during the pandemic.

## 5. Conclusions

At the state level, Khartoum State was the most benefited state from the healthcare services of Imperial Hospital. At a locality level, Khartoum locality was the most benefited one. That might be related to the urbanization of the population and the ease of access to healthcare services. Furthermore, patients from different states of Sudan had traveled to reach Imperial Hospital for medical care. This issue needs to be addressed by concerned authorities.

## 6. Recommendations

Similar studies must be conducted to assess the extent of the healthcare system during the pandemic in Sudan, in both private and governmental sectors. This will allow specialists to locate the areas in need of healthcare centers and COVID-19 care services.

## Figures and Tables

**Figure 1:** COVID-19 hospitalized cases at Imperial Hospital across the states of Sudan (*n* = 188).

**Figure 2:** Extent of healthcare services of Imperial Hospital across Khartoum State (*n* = 167), a hotspot analysis of COVID-19 cases across the localities of Khartoum State.

**Figure 3:** Hotspot analysis of COVID-19 cases covered by Imperial Hospital services. Population and cases in Khartoum State at localities level.

**Figure 4:** Population and cases across the localities of Khartoum State.

**Figure 5:** Radius of Imperial Healthcare Services for COVID-19 patients across Khartoum State. Risk prediction map for COVID-19 in Khartoum State.

**Figure 6:** COVID-19 risk map of Khartoum State.

## Data Availability

All supporting data are available from the corresponding author on reasonable request.

## Abbreviations

GIS: Geographic information system
RT-PCR: Reverse transcriptase-polymerase chain reaction
LAT: Latitude
LON: Longitude.
